# The Effect of Business Cycles on Health Expenditure: A Story of Income Inequality in China

**DOI:** 10.3389/fpubh.2021.653480

**Published:** 2021-03-18

**Authors:** Xiaohong Pu, Ming Zeng, Yaling Luo

**Affiliations:** School of Public Administration, Sichuan University, Chengdu, China

**Keywords:** business cycles, health expenditure, income inequality, financial crisis, population health

## Abstract

Using the panel data of 31 regions in China from 2002 to 2018, this study aims to investigate the effect of business cycles on health expenditure from the role of income inequality. We find that health expenditure experiences a change from pro-cyclical to counter-cyclical with business cycles. Specifically, business cycles have a different influence on health expenditure before and after the financial crisis in 2008. Our findings also show that income inequality can moderate the impact of business cycles on health expenditure in China. More importantly, the role of income inequality in the above issue varies from different regions. We conclude that the government should try to take active steps to control health expenditure by decreasing income inequality.

## Introduction

During the economic downturn caused by COVID-19, the relationship between business cycles and health issues has again attracted the attention of academics (1). In fact, health expenditure is directly related to residents' health level and living standard. According to China's National Statistics Bureau (2), the total health expenditure has increased from 5,709.03 billion RMB in 2002 to 59,121.91 billion RMB in 2018, and the share of health expenditure in the gross domestic product (GDP) has fluctuated from 4.76% in 2002 to 6.57% in 2018. Figure 1 shows the trend of business cycles and health expenditure in China during 2002–2018^1^. As can be seen from the figure, the trend of health expenditure is opposed to that of business cycles during 2002–2018. It indicates that the faster China's economic development is, the smaller the share of health expenditure will be. We can generally conclude that health expenditure is counter-cyclical with business cycles in China during 2002–2018.

**Figure 1:** The trend of business cycles and health expenditure in China during 2002–2018.

The impact of business cycles on health expenditure has always been controversial among academics. Some studies have widely verified that health expenditure is pro-cyclical with business cycles (3–5). That is, economic booms lead to more health expenditure, while recessions have a negative effect on health expenditure. The studies also have stated that there are many reasons for the above situations, such as medical affordability (6–8) and environmental quality (9–13). However, some scholars have claimed that the link between business cycles and health expenditure varies with the income level. For example, health expenditure is counter-cyclical with business cycles in low-income countries (14, 15). Besides, health expenditure is directly related to population health, and the mixed relationship between business cycles and population health can make this issue more complicated (16–26). Many interesting findings of business cycles and health expenditure have been made, but rare literature focuses on this issue in China from the role of income inequality.

In this study, we attempt to investigate how business cycles affect health expenditure in China, and we also extend the understanding of the above link from the role of income inequality. We investigate the issue motivated by the following considerations. China is the largest and fastest-growing emerging market in the world, and it is a very exciting subject to study because of its culture and history (27, 28). According to the *World Economic Outlook* issued by the International Monetary Fund (IMF) in October 2020, China is likely to be the only economy to achieve positive growth in 2020, at about 1.9 percent, and is expected to contribute about a third of the global economy in 2021 (29). Hence, it is of theoretical and practical significance for academics to investigate the effect of business cycles on health expenditure in China.

We explore the dynamic effect of business cycles on health expenditure in China using the individual fixed-effect model. Among them, business cycles are measured by the growth rate of GDP, and health expenditure is measured by outpatient expenditure. More importantly, we investigate the role of income inequality in the dynamic effect by introducing a moderator model and explore its heterogeneity from the perspectives of regional differences. We also take some robust tests for our findings.

We make several interesting findings. First, there is a dynamic change in the impact of business cycles on health expenditure in China. That is, health expenditure in China changes from pro-cyclical to counter-cyclical with business cycles. Second, income inequality can weaken the reduction effects of business cycles on health expenditure. Third, our findings show that the above relationships vary with different regions. Finally, we conduct a series of robustness tests and the results further show that our findings are robust.

This study fills some existing gaps in the literature on business cycles and health expenditure. The main novelties and contributions of our study are listed as follows: First, to our best knowledge, this study may be the first research to analyze this issue in China. There are some differences between developed countries and emerging countries in the impact of business cycles on health expenditure. Previous studies on this issue lack research on emerging economies, and this study has extraordinary significance for easing that shortage. Second, we extend the understanding of the link between business cycles and health expenditure by investigating the role of income inequality. Income inequality can harm residents' health by bringing more pressure and anxiety into society, resulting in an increase of health expenditure. Because rare studies place particular emphasis on the role of income inequality in this issue, this study enlarges the research vision on the impact of business cycles on health expenditure.

This study is organized as follows. Literature Review section provides a summary and review of the existing literature. Models and Data section mainly describes the research hypotheses, data, and empirical models used in the study. Results and Discussions section presents the empirical results, and Further Analysis section discusses the results in more detail. The final section summarizes our main conclusions and policy implications.

## Literature Review

Previous studies have conducted a series of research on the relationship between business cycles and health expenditure from different perspectives. A basic consensus has been reached that health expenditure can accelerate economic growth and lead to economic booms by improving population health and accumulating human capital (30–34). While the impact of business cycles on health expenditure remains unclear and inconclusive. Some literature claims that health expenditure is pro-cyclical with business cycles (3–5). For example, Bedir (6), Payandeh et al. (7), and Kumar et al. (8) point out that the increase of residents' disposable income during boom periods guarantees their ability to pay for medical needs, resulting in more increases in health expenditure. Badulescu et al. (9), Haseeb et al. (10), Wang et al. (11), Mujtaba and Shahzad (12), and Urhie et al. (13) claim that economic booms are associated with worse environmental quality, which in turn results in lower population health and more expenditure on health.

However, other studies have shown some different results. Some scholars claim that in low-income countries, health expenditure is counter-cyclical with business cycles. That is, residents decrease their health expenditure in good times, while they increase health expenditure in the doldrums. For instance, Rana et al. (14) state that the effect of business cycles on health expenditure varies with income levels. They also point out that in low-income countries, residents decrease health expenditure during economic booms. Jakovljevic et al. (15) explore the differences related to this issue between developed countries and emerging countries and reach similar conclusions. That is, economic booms have a positive impact on health expenditure in developed countries while they negatively affect health expenditure in emerging countries. Universal healthcare and the aging population are two important factors contributing to these differences.

Besides, business cycles can affect health expenditure through population health. Obviously, the residents' health plays a non-negligible role in the health expenditure, because health level is directly related to the needs of medical services. The effect of business cycles on population health is mixed. Some literature indicates that the impact of business cycles on population health is pro-cyclical (16–20). In contrast, some studies suggest that population health is counter-cyclical with business cycles (21–24). For example, Lam and Pierard (25) and Lee and Kim (26) find that population health has undergone a dramatic change from counter-cyclical to pro-cyclical in the United States and South Korea, respectively.

Many interesting results have been found on the above issues, but there are still some gaps needed to be filled. First, most studies have discussed the relationship between business cycles and health expenditure in developed countries such as the United States and Europe (4, 9), while limited studies have paid attention to this issue in emerging markets (6, 20). However, there are some differences between emerging economies and developed economies in political, economic, and cultural aspects (35–37), and business cycles may have different effects on health expenditure. Second, most studies have discussed the counter-cyclical or pro-cyclical effects of business cycles on health expenditure from the following perspectives, such as medical affordability (6–8), environmental quality (9–13), universal healthcare (15), aging population (15), and population health (16–26). However, we find nearly no related studies that explore the above relationship from the role of income inequality. Income inequality can affect population health in the following ways: consumption capacity (38–40), psychological state (41–43), and social relations (44–46). Hence, income inequality may influence the effect of business cycles on health expenditure. Finally, so far, little literature focuses on the change of the impact of business cycles on health expenditure. The 2008 financial crisis has brought about major changes in the world economy (15), which may affect the relationship between business cycles and health expenditure.

## Models and Data

### Research Hypotheses

China has paid more and more attention to environmental protection in recent years, as the environmental pollution caused by rapid economic growth has become more serious. Health problems caused by environmental pollution increase health expenditure (47–49). During the 13th Five-Year Plan period, China has made remarkable achievements in improving environmental quality (50). The achievement can decrease the health expenditure caused by environmental pollution during the economic booms. Besides, the residents' health level is insignificantly improved with the development of China (51–53). Better health may well mean lower health expenditure. Due to the improvement of environmental quality and population health, we propose the following hypothesis:

H1: Health expenditure experiences a pro-cyclical to counter-cyclical change with business cycles.

Many related studies have verified that income inequality can adversely affect population health (38–46). Economic booms can benefit population health by guaranteeing the residents more material goods and medical goods. But, the beneficial effects of economic booms on population health will be offset by the unequal distribution of national income. Due to the close ties between population health and health expenditure, we propose the following hypothesis:

H2: Income inequality can affect the relationship between business cycles and health expenditure.

### Data

This study aims to investigate the impact of business cycles on health expenditure in China from the perspective of income inequality using the data of 31 regions in China from 2002 to 2018. These regions include Beijing, Tianjin, Hebei, Shanxi, Inner Mongolia, Liaoning, Jilin, Heilongjiang, Shanghai, Jiangsu, Zhejiang, Anhui, Fujian, Jiangxi, Shandong, Henan, Hubei, Hunan, Guangdong, Guangxi, Hainan, Chongqing, Sichuan, Guizhou, Yunnan, Tibet, Shaanxi, Gansu, Qinghai, Ningxia, and Xinjiang. The data of outpatient expenditure, number of outpatient visits, hospitalization expenditure, and number of hospitalization are collected from the Chinese Health Statistical Yearbook 2003–2019 (54). The data of GDP and per capita disposable income of urban and rural residents in different regions are collected from the Chinese Statistical Yearbook 2003–2019 (55). The environmental quality data in different regions during 2002–2018 are from Dalhousie University Atmospheric Composition Analysis Group (56). The other data, such as aging ratio, urbanization level, and gender ratio, are collected from the Chinese Population & Employment Statistical Yearbook 2003–2019 (57).

### Variables

(1) Health Expenditure (*exp_out*)

Referring to the related research (58–60), we use outpatient expenditure (*exp*_*out*) to measure health expenditure. It is measured by the ratio of the total outpatient expenditure to the total number of outpatient visits. Besides, we also apply the following proxy variables to conduct robust tests: number of outpatient visits (num_out), hospitalization expenditure (*exp*_*hos*), and number of hospitalization (*num*_*hos*). The number of outpatient visits is measured by the natural logarithm of the total number of outpatient visits. Hospitalization expenditure is expressed as the ratio of the total hospitalization expenditure to the total number of hospitalization. The number of hospitalization is measured by the natural logarithm of the total number of hospitalization.

(2) Business Cycles (*Bus_cycles*)

The existing literature mainly uses the unemployment rate (22, 23) and the GDP growth rate (20, 25, 61, 62) to measure business cycles. Since there is a large deviation between the reported unemployment rate and the actual unemployment rate in China, the conclusions may be biased. Hence, we use the GDP growth rate to measure business cycles.

(3) Income Inequality (*inequality*)

Income inequality is defined as the income gap between urban and rural areas, which is measured by the ratio of the per capita disposable income of urban residents to that of rural residents.

(4) Control Variables

As we all know, health expenditure is affected not only by the above independent variables but also by many others, such as environmental quality and demographic characteristics. Referring to the existing studies (3, 15, 62), we control the following variables: environmental quality (*environment*), aging ratio (*aging*), urbanization level (*urban*), and gender ratio (*gender*).

The above variables and their definitions are presented in Table 1, and their descriptive statistics are shown in Table 2.

**Table 1:** Description of the variables.

**Types**	**Variables**	**Symbols**	**Definitions**
Dependent variables	Outpatient expenditure	*exp_out*	The ratio of the total outpatient expenditure to the total number of outpatient visits.
	Number of outpatient visits	*num_out*	The natural logarithm of the total number of outpatient visits.
	Hospitalization expenditure	*exp_hos*	The ratio of the total hospitalization expenditure to the total number of hospitalization.
	Number of hospitalization	*num_hos*	The natural logarithm of the total number of hospitalization.
Independent variables	Business cycles	*Bus_cycles*	The real annual growth rate of GDP.
	Income inequality	*inequality*	The ratio of the per capita disposable income of urban residents to that of rural residents.
Control variables	Environmental quality	*environment*	The natural logarithm of the average PM_2.5_ concentrations.
	Aging ratio	*aging*	The proportion of the residents aged 65 and over to the total population.
	Urbanization level	*urban*	The ratio of the urban population to the total population.
	Gender ratio	*gender*	The ratio of the number of men to the total population.

**Table 2:** Descriptive statistics.

**Variables**	**Obs**	**Mean**	**S.D**.	**Min**	**Median**	**Max**
*exp_out*	527	5.0243	0.4479	3.2347	5.0486	6.3004
*num_out*	527	17.7014	0.9693	14.5140	17.7942	19.7420
*exp_hos*	527	8.6626	0.4614	7.5492	8.6818	10.0265
*num_hos*	527	14.6200	1.0555	10.7110	14.7608	16.4969
*Bus_cycles*	527	0.1374	0.0117	−0.224	0.1238	0.6077
*inequality*	527	2.9065	0.6044	1.8451	2.7819	5.6048
*environment*	527	3.4595	0.5791	1.4110	3.5732	4.4262
*aging*	527	0.0920	0.0211	0.0476	0.0892	0.1638
*urban*	527	0.5041	0.1539	0.2022	0.4931	0.9418
*gender*	527	0.5105	0.0090	0.4798	0.5100	0.5463

### Method

Referring to the related research (3, 15, 63), our regression model is set as follows:

(1) $$\begin{array}{l} Y_{it}=\alpha +\beta_{1}Bus\_cycles_{it}+\gamma_{1}environment_{it}+\gamma_{2}aging_{it}\\ \;+\gamma_{3}urban_{it}+\gamma_{4}gender_{it}+u_{i}+\varepsilon_{it} \end{array}$$

where *Y* is the dependent variable of health expenditure; *Bus_cycles* is the independent variable of business cycles; *environment, aging, urban*, and *gender* are the control variables; α denotes the intercept item; β_1_ denotes the coefficient of business cycles; γ denotes the coefficient of the control variables; *i* represents the region and *t* represents year; *u*_*i*_ is the individual fixed-effect; and ε_*it*_ is a normally distributed random error vector.

If β_1_ is >0, it indicates that the faster China's economic development is, the higher the health expenditure will be. In other words, health expenditure has a pro-cyclical relationship with business cycles. In contrast, if β_1_ is <0, it means that the faster China's economic development is, the lower the health expenditure will be. That is, health expenditure is counter-cyclical with business cycles. Furthermore, if β_1_ changes from >0 to <0 at a given year, it indicates that health expenditure undergoes a pro-cyclical to counter-cyclical change in China.

To further explore the mechanism of income inequality on the relationship between business cycles and health expenditure, we introduce *inequality* and the interaction term of the form *Bus_cycles* × *inequality* into Model (1). Model (2) is constructed as follows:

(2) $$\begin{array}{l} Y_{it}=\alpha +\beta_{1}Bus\text{\_}cycles_{it}+\beta_{2}inequality\\ \;+\beta_{3}Bus\text{\_}cycles\times inequality+\gamma_{1}environment_{it}\\ \;+\gamma_{2}aging_{it}\;+\gamma_{3}urban_{it}+\gamma_{4}gender_{it}\text{+}u_{i}+\varepsilon_{it} \end{array}$$

where β_2_ represents the coefficient of income inequality and β_3_ represents the coefficient of interactive item between income inequality and business cycles.

If β_3_ is >0, it indicates that when *inequality* is bigger, the increase of *Bus_cycles* will induce bigger *Y*. That is, when the distribution of income is more unequal in China, economic development will bring more health expenditure. Hence, income inequality can strengthen the increase effect of business cycles on health expenditure when β_1_ is >0, and it weakens the reduction effect when β_1_ is <0. In contrast, if β_3_ is <0 and β_1_ is >0, it means that income inequality can weaken the increase effect. While when both β_1_ and β_3_ are smaller than 0, it means that income inequality can strengthen the reduction effect.

## Results and Discussions

In this section, we first examine the impact of business cycles on health expenditure by using Model (1). Then, we explore the effect of income inequality on the relationship between business cycles and health expenditure by using Model (2). Finally, we examine whether the above issues vary with the different regions.

### The Impact of Business Cycles on Health Expenditure

The estimated results are reported in Table 3. Among them, columns (1) and (2) are the results of the samples during 2002–2018, columns (3) and (4) are the results of the samples during 2002–2008, and columns (5) and (6) are the results of the samples during 2008–2018.

**Table 3:** Estimation results of business cycles and health expenditure.

**Variables**	**Samples 2002**–**2018**		**Samples 2002**–**2008**		**Samples 2008**–**2018**	
	**(1)**	**(2)**	**(3)**	**(4)**	**(5)**	**(6)**
*Bus_cycles*	−2.400^***^ (−12.19)	−0.662^***^ (−4.82)	1.353^***^ (8.26)	0.818^***^ (5.32)	−2.149^***^ (−14.11)	−0.502^***^ (−4.89)
*environment*		0.073 (1.31)		0.148^**^ (2.34)		−0.049 (−1.18)
*aging*		6.641^***^ (7.24)		8.103^***^ (6.24)		1.366^**^ (2.10)
*urban*		3.289^***^ (19.09)		0.617^***^ (3.18)		4.206^***^ (21.81)
*gender*		9.331^***^ (7.01)		−0.679 (−0.30)		2.515^***^ (3.11)
_cons	5.359^***^ (173.76)	−2.191^***^ (−2.97)	4.426^***^ (142.84)	3.366 (2.71)	5.495^***^ (263.93)	1.765^***^ (3.61)
Individual FE	Yes	Yes	Yes	Yes	Yes	Yes
*N*	527	527	217	217	341	341
*R*^2^	0.1487	0.6518	0.0543	0.6565	0.2271	0.6495

*** *1% significance level*,

** *5% significance level. The t statistics are in the brackets*.

When we use the samples from 2002 to 2018, the coefficients of *Bus_cycles* in columns (1) and (2) are significantly negative at the 1% level. It indicates that business cycles in China have a significantly adverse impact on health expenditure during 2002–2018. That is, the faster China's economic development is, the lower the health expenditure will be. The improved living conditions of residents during economic booms make them relatively healthy, which reduces the likelihood that they will need medical resources. Hence, health expenditure decreases during economic booms while it increases in recessions. In a word, health expenditure is counter-cyclical with business cycles in China.

Second, we divide the samples into two parts (before and after the 2008 financial crisis) to further explore whether health expenditure experiences a pro-cyclical to counter-cyclical change with business cycles in China. The 2008 financial crisis has had a profound impact on world economic development (63–65), which may affect the relationship between business cycles and health expenditure (66, 67). Hence, we divide the samples into samples 2002–2008 and samples 2008–2018, and the estimation results are given in columns (3)–(6). The coefficients of *Bus_cycles* in columns (3) and (4) are significantly positive at the 1% level. It indicates that economic booms lead to more health expenditure, and health expenditure is pro-cyclical with business cycles in China before the 2008 financial crisis. However, the coefficients of *Bus_cycles* in columns (5) and (6) are significantly negative at the 1% level. It suggests that economic booms lead to fewer health expenditure, and health expenditure is counter-cyclical with business cycles in China after the 2008 financial crisis. In a word, health expenditure experiences a pro-cyclical to counter-cyclical change with business cycles in China from 2002 to 2018. Our conclusions support hypothesis 1. The improvement of population health decreases the health expenditure during economic booms, and it may be an important factor promoting this change of health expenditure.

For all the control variables, the coefficient of *environment* is only positive at the 5% significance level for the samples 2002–2008, which shows that the worse environmental quality has a significant increased impact on health expenditure before the 2008 financial crisis. All the coefficients of *aging* in columns (2), (4), and (6) are significantly positive at the 5% level, which indicates that population aging can increase health expenditure. The coefficients of *urban* are also positive and significant at the 1% level, indicating that the health expenditure in urban areas is higher than that in rural areas. All the coefficients of *gender* are significantly positive at the 1% level except for the one in column (4), which indicates that men have greater health expenditure than women in China after the 2008 financial crisis.

### The Moderating Effect of Income Inequality

In this subsection, we adopt Model (2) to explore the moderating effect of income inequality. The empirical results are presented in Table 4. Among them, column (1) is the results of the samples during 2002–2018, column (2) is the results of the samples during 2002–2008, and column (3) is the results of the samples during 2008–2018.

**Table 4:** Estimation results of the moderating effect of income inequality.

**Variables**	**Samples 2002–2018**	**Samples 2002–2008**	**Samples 2008–2018**
	**(1)**	**(2)**	**(3)**
*Bus_cycles*	−2.164^***^ (−3.61)	−0.964 (−1.42)	−1.552^***^ (−3.13)
*inequality*	−0.544^***^ (−12.03)	−0.327^***^ (−4.72)	−0.251^***^ (−5.40)
*Bus_cycles* × *inequality*	0.647^***^ (3.16)	0.609^***^ (2.69)	0.385^**^ (2.29)
*environment*	0.151^***^ (3.29)	0.140^**^ (2.33)	−0.048 (−1.20)
*aging*	4.958^***^ (6.44)	7.762^***^ (6.24)	1.656^**^ (2.53)
*urban*	2.523^***^ (16.84)	0.955^***^ (4.66)	3.123^***^ (11.00)
*gender*	5.584^***^ (4.93)	−1.786 (−0.81)	1.958^**^ (2.46)
_cons	1.518^**^ (2.24)	4.831^***^ (3.95)	3.300^***^ (5.97)
Individual FE	Yes	Yes	Yes
*N*	527	217	341
*R*^2^	0.6482	0.7074	0.6817

*** *1% significance level*,

** *5% significance level. The t statistics are in the brackets*.

For the results of the whole sample in column (1), the coefficient of *Bus_cycles* is significantly negative at the 1% level, suggesting that economic booms decrease the health expenditure. These results are consistent with the above conclusions and further verify hypothesis 1. The coefficient of the interaction term *Bus_cycles* × *inequality* is significantly positive at the 1% level, which suggests that income inequality can weaken the negative impact of business cycles on health expenditure in China. The possible reason is that the income elasticity of health expenditure for the rich is higher than that for the poor, and income inequality can increase the rich's health expenditure and induce a minor decrease for the poor, resulting in an increase of the total health expenditure. Our findings verify hypothesis 2.

When we consider the 2008 financial crisis, the results show that the coefficients of *Bus_cycles* × *inequality* are still significant and positive at the 5% level. They indicate that income inequality can weaken the reduction effects of economic booms on health expenditure. These results are consistent with the above findings. Hence, the moderating effect of income inequality remains stable during the study period in China.

### Heterogeneity Analysis for Different Regions

In this subsection, we further investigate the heterogeneity of different regions, and the estimation results are reported in Table 5. Among them, columns (1) and (2) are the results for the eastern regions, columns (3) and (4) are the results for the central regions, and columns (5) and (6) are the results for the western regions. Columns (1), (3), and (5) are the results for Model (1), and columns (2), (4), and (6) are the results for Model (2). All the columns are the results of the samples during 2002–2018.

**Table 5:** Estimation results of different regions.

**Variables**	**Eastern regions**		**Central regions**		**Western regions**	
	**(1)**	**(2)**	**(3)**	**(4)**	**(5)**	**(6)**
*Bus_cycles*	−0.721^***^ (−4.25)	−1.377 (−0.94)	−0.547^***^ (−3.35)	−1.173 (−0.86)	−0.646^**^ (−2.37)	−4.284^***^ (−3.17)
*inequality*		0.072 (0.63)		−0.340^***^ (−3.79)		−0.688^***^ (−9.43)
*Bus_cycles* × *inequality*		0.240 (0.42)		0.298 (0.62)		1.284^***^ (3.19)
Control variables	Yes	Yes	Yes	Yes	Yes	Yes
Individual FE	Yes	Yes	Yes	Yes	Yes	Yes
*N*	187	187	136	136	204	204
*R*^2^	0.6199	0.6050	0.8156	0.8005	0.5976	0.6971

*** *1% significance level*,

** *5% significance level. The t statistics are in the brackets*.

All the coefficients of *Bus_cycles* in columns (1), (3), and (5) are significantly negative at the 5% level, which indicates health expenditure is counter-cyclical with business cycles in the three regions of China. The coefficient of the interaction term *Bus_cycles* × *inequality* is significantly positive at the 1% level in column (6), while it does not exceed the 10% significance level in columns (2) or (4). These results suggest that the role of income inequality in the relationship between business cycles and health expenditure varies from the different regions. Only in the western regions, income inequality can moderate the impact of business cycles on health expenditure.

## Further Analysis

### Endogenous Test

The above findings show that business cycles can affect health expenditure, but there may be reverse causality between business cycles and health expenditure. Although we control some important variables that can affect health expenditure in the empirical analysis, it is impossible to completely rule out endogeneity. Therefore, we use the instrumental variable method (IV) to partly control endogenous problems. We take the growth rate of GDP lag by one stage as the instrumental variable for business cycles and estimate Model (1) with the two-stage least square method (2SLS). The estimation results are reported in Table 6. Among them, columns (1)–(3) are the results of the samples during 2002–2018, the samples during 2002–2008, and the samples during 2008–2018, respectively. The coefficient of *Bus_cycles* in column (1) is significantly negative at the 5% level, which indicates health expenditure in China is counter-cyclical with business cycles during 2002–2018. The coefficient of *Bus_cycles* in column (2) is significantly positive, while the one in column (3) is significantly negative. It indicates that health expenditure in China experiences a pro-cyclical to counter-cyclical change with business cycles during 2002–2018. These results are consistent with the above findings, which further verifies our conclusions.

**Table 6:** Estimation results of the endogenous test.

**Variables**	**Samples 2002–2018**	**Samples 2002–2008**	**Samples 2008–2018**
	**(1)**	**(2)**	**(3)**
*Bus_cycles*	−0.905^**^ (−2.46)	7.403^**^ (2.01)	−1.990^**^ (−2.44)
Control variables	Yes	Yes	Yes
Individual FE	Yes	Yes	Yes
*N*	527	217	341
*R*^2^	0.6567	0.0332	0.6674

** *5% significance level. The z values are in the brackets*.

### Robustness Test

To further make sure the robustness of the above conclusions, we replace the variable of health expenditure with number of outpatient visits (*num_out*), hospitalization expenditure (*exp_hos*), and number of hospitalization (*num_hos*). The estimation results of the robustness tests are reported in Table 7. Among them, columns (1), (3), and (5) are the results for Model (1), and columns (2), (4), and (6) are the results for Model (2). Columns (1) and (2) are the results of the samples during 2002–2018, columns (3) and (4) are the results of the samples during 2002–2008, and columns (5) and (6) are the results of the samples during 2008–2018. The results are all consistent with the previous results, indicating that our findings remain robust using the different proxy variables.

**Table 7:** Estimation results of the robustness tests.

**Variables**	**Samples 2002**–**2018**		**Samples 2002**–**2008**		**Samples 2008**–**2018**	
	**(1)**	**(2)**	**(3)**	**(4)**	**(5)**	**(6)**
**Panel A: The dependent variable is number of outpatient visits (*****num*****_*****out*****)**.						
*Bus_cycles*	−0.881^***^ (−6.85)	−3.444^***^ (−5.91)	0.422^***^ (2.73)	−1.096 (−1.56)	−0.442^***^ (−5.32)	−1.649^***^ (−4.03)
*inequality*		−0.525^***^ (−11.93)		−0.235^***^ (−3.28)		−0.152^***^ (−3.95)
*Bus_cycles* × *inequality*		0.993^***^ (4.99)		0.519^**^ (2.22)		0.428^***^ (3.08)
*R*^2^	0.3115	0.3587	0.4062	0.3991	0.2636	0.2703
**Panel B: The dependent variable is hospitalization expenditure (*****exp*****_*****hos*****)**.						
*Bus_cycles*	−0.630^***^ (−4.88)	−2.684^***^ (−4.33)	0.815^***^ (5.22)	0.419 (0.06)	−0.436^***^ (−4.75)	−1.985^***^ (−4.48)
*Inequality*		−0.432^***^ (−9.21)		−0.158^**^ (−2.15)		−0.221^***^ (−5.32)
*Bus_cycles × inequality*		0.799^***^ (3.77)		0.264(1.10)		0.551^***^ (3.66)
*R*^2^	0.7134	0.6896	0.6621	0.6812	0.8275	0.8466
**Panel C: The dependent variable is number of hospitalization (*****num*****_*****hos*****)**.						
*Bus_cycles*	−0.894^***^ (−4.83)	−3.005^***^ (−3.72)	1.001^***^ (4.58)	−1.994^**^ (−2.05)	−0.551^***^ (−4.86)	−1.413^**^ (−2.56)
*inequality*		−0.741^***^ (−12.15)		−0.413^***^ (−4.16)		−0.244^***^ (−4.71)
*Bus_cycles × inequality*		0.902^***^ (3.28)		1.023^***^ (3.15)		0.320* (1.71)
*R*^2^	0.1720	0.2164	0.2454	0.2356	0.0635	0.0786
Control Variables	Yes	Yes	Yes	Yes	Yes	Yes
Individual FE	Yes	Yes	Yes	Yes	Yes	Yes
*N*	527	527	217	217	341	341

*** *1% significance level*,

** *5% significance level. The t statistics are in the brackets*.

## Conclusions

Using the panel data of 31 regions in China from 2002 to 2018, this study aims to examine the impact of business cycles on health expenditure from the role of income inequality. The main conclusions drawn are as follows:

1. The impact of business cycles (represented by the growth rate of GDP) on health expenditure (represented by outpatient expenditure) experiences a change from pro-cyclical to counter-cyclical. Specifically, economic booms increase the health expenditure before the 2008 financial crisis, while they have a negative impact on health expenditure after the 2008 financial crisis. The conclusions are robust when we use number of outpatient visits, hospitalization expenditure, and number of hospitalization as the proxy variables of health expenditure.
2. Income inequality can moderate the impact of business cycles on health expenditure in China. In practical terms, income inequality would increase the health expenditure incurred by economic booms. In other words, income inequality will weaken the reduction effects of business cycles on health expenditure.
3. By exploring the heterogeneity of regions, our findings show that health expenditure is counter-cyclical with business cycles in the eastern regions, the central regions, and the western regions. However, only in the western regions income inequality can affect the relationship between business cycles and health expenditure.

According to the conclusions above, we have drawn some policy implications. First, health expenditure is counter-cyclical with business cycles in China, which indicates economic recessions induce more health expenditure. Hence, policymakers should be more forceful in times of economic recessions than in economic expansion periods. Second, the reduction effects on health expenditure in economic booms can be weakened by income inequality. Great attention must be paid to income distribution when the government develops the economy, especially in the western regions. To control health expenditure, the government should take active steps to narrow the income gap among different regions and residents. For example, the government should deepen the reform of the income distribution system and improve the social security system.

Finally, we put forward some future research topics. First, it is hoped that this study will spur more theoretical and empirical research on business cycles, population health, and health expenditure. Scholars have made much effort to explore the relationship between business cycles and the other two topics, but there is little existing research on these three topics. Second, academics should further analyze the mechanism by which business cycles affect health expenditure. Our study finds that health expenditure decreases in booms while it increases in recessions. However, the influence mechanism still needs further studies. Third, health expenditure experiences pro-cyclical to counter-cyclical with business cycles in China, but the reasons behind this phenomenon are unclear. Further studies are still needed to offer more explanations for the above conclusions.

## Data Availability Statement

The original contributions presented in the study are included in the article/supplementary material, further inquiries can be directed to the corresponding author.

## Author Contributions

XP: conceptualization, writing—original draft, and software. MZ: information collection, literature search, and writing—original draft. YL: writing—reviewing and editing and supervision. All authors contributed to the article and approved the submitted version.

## Conflict of Interest

The authors declare that the research was conducted in the absence of any commercial or financial relationships that could be construed as a potential conflict of interest.

## Footnotes

^1^The business cycles are expressed by the growth rate of GDP per capita, and the health expenditure is expressed by the growth rate of the share of health expenditure.
